# Microstructure and Mechanical Properties of Gradient Nanostructured Q345 Steel Prepared by Ultrasonic Severe Surface Rolling

**DOI:** 10.1155/2023/7705844

**Published:** 2023-04-17

**Authors:** Chao Ge, Weilong Meng, Handui Feng, Muchun Cui, Lei Dong, Tianfeng Miao, Yantong Huo, Jiemin Wu, Jing Han

**Affiliations:** ^1^Xuzhou XCMG Mining Machinery Co. LTD, Xuzhou 221000, China; ^2^CUMT-XCMG Mining Intelligent Equipment Technology Research Institute, China University of Mining and Technology, Xuzhou 221116, China; ^3^School of Mechanical and Electrical Engineering, China University of Mining and Technology, Xuzhou 221116, China

## Abstract

In this work, ultrasonic severe surface rolling (USSR), a new surface nanocrystallization technique, is used to prepare gradient nanostructure (GNS) on the commercial Q345 structural steel. The microstructure of the GNS surface layer is characterized by employing EBSD and TEM, and the result indicates that a nanoscale substructure is formed at the topmost surface layer. The substructures are composed of subgrains and dislocation cells and have an average size of 309.4 nm. The GNS surface layer after USSR processing for one pass has a thickness of approximately 300 *μ*m. The uniaxial tensile measurement indicates that the yield strength of the USSR sample improves by 25.1% compared to the as-received sample with slightly decreased ductility. The nanoscale substructure, refined grains, high density of dislocations, and hetero-deformation-induced strengthening are identified as responsible for the enhanced strength. This study provides a feasible approach to improving the mechanical properties of structural steel for wide applications.

## 1. Introduction

As common low-alloy steel, Chinese standard Q345 steel exhibits medium strength, good plasticity, and good weldability and is thus widely used in engineering machinery, ships, bridges, steel buildings, pressure vessels, offshore platforms, and other applications. Q345 steel is similar to ASTM A572 grade 50 steel in the U.S. and European standard S355 steel in Europe in terms of its mechanical properties. However, improved strength without visibly sacrificed plasticity is needed for Q345 steel to meet the high-strength requirement of key components or local regions of key components.

Constructing gradient nanostructures (GNSs) have been proven to be a good strategy for enhancing the mechanical properties of metals and alloys inspired by nature [1, 2]. Over the past two decades, this strategy has been successfully applied in almost all types of structural metallic materials [3–7], such as Cu and Cu alloys [8, 9], Mg alloys [10, 11], and Ti alloys [12, 13]. Several methods have been developed to prepare the gradient nanostructure, such as surface mechanical grinding treatment (SMGT) [3], surface mechanical attrition treatment (SMAT) [14], surface mechanical rolling treatment (SMRT) [15], laser shock peening (LSP) [16], ultrasonic surface rolling (USR), or ultrasonic nanocrystalline surface modification (UNSM) [17–20]. Among these, USR is an effective and easy-to-operate method that has been applied in several steels. Ye et al. [21] applied USR on a 40 Cr (a medium carbon alloy steel) and generated a GNS with a grain size of 3-7 nm in the topmost surface layer, leading to a 52.6% improvement in surface microhardness. However, the strength and plasticity of the GNS 40 Cr were not involved. Liu et al. [22] found that UNSM induced a GNS in AISI 304 stainless steel as well as gradient martensite content, and the average grain size in the topmost surface layer was 4.1 nm. After UNSM, the strength of AISI 304 stainless steel improved from 340 MPa to 630 MPa while still preserving high ductility. Recently, a modified USR method, called ultrasonic severe surface rolling (USSR), was proposed by Han et al. to obtain a superior gradient surface layer [10]. USSR produces a high strain rate of approximately 10^5^/s, which is much higher than many other techniques of preparing GNSs, such as SMAT (10^2^~10^3^/s), SMGT (10^3^~10^4^/s), and SMRT (10^3^~10^4^/s) [2, 10]. USSR applies a large static force on the treated surface for forming a large gradient plastic strain. The large strain and high strain rate enable a thick gradient nanostructure and superior mechanical properties for various metals and alloys. Also, USSR synchronously prepares a high-quality surface with low roughness and few processing defects. Our previous work found that USSR forms a gradient structured surface layer with a thickness of ~1 mm in the selective laser melted (SLM) 316L stainless steel, endowing the steel with improved strength without a significant loss in ductility as well as enhanced corrosion resistance in NaCl solution [22, 23].

In the present study, USSR is applied to commercial Q345 structural steel to improve its mechanical properties by forming a GNS. The detailed microstructure of the USSR sample was characterized by electron backscatter diffraction (EBSD) and transmission electron microscopy (TEM), and an attempt was made to link the microstructure to the improved mechanical properties.

## 2. Methods

A commercial hot-rolled Q345 steel plate was used as the initial material. The as-received plate was machined into sheets 50 mm × 25 mm × 4 mm in size and then processed by one pass of USSR on two parallel surfaces at room temperature. The process parameters can be found in our previous work [22], but a relatively small static force of 600 N was applied in this study. During USSR processing, the cutting fluid was used to cool and reduce friction.

The microstructure of the as-received sample was characterized by an optical microscope (OM), scanning electron microscopy (SEM, Hitachi Regulus8100), and EBSD (Oxford Instrument C-Nano). The depth-dependent microstructure of the USSR sample was observed by cross-section EBSD observation. The microstructure of the topmost surface layer was further characterized by TEM (FEI Talos F200X).

The microhardness profile along the depth of the as-received and USSR samples was measured by a Vickers hardness tester. The applied load and duration time were 0.49 N and 10 s, respectively. The mechanical properties were examined through the uniaxial tensile test at room temperature at a speed of 0.5 mm/min. The tensile specimens had a gauge length of 7.5 mm and original width of 2 mm.

## 3. Results

The OM and SEM images indicate that the as-received sample is composed of ferrite and a small amount of pearlite, as indicated in Figure 1. The EBSD inverse pole figure (IPF) and bond contrast (BC) maps show that the ferrite has an average grain size of 5.6 *μ*m and contains a few low angle grain boundaries (LAGBs), as shown in Figure 2. The high kernel average misorientation (KAM) values in some grains imply that the as-received sample involves some lattice defects (Figure 2(d)), most of which are dislocations in this material.

Figure 3 presents the cross-sectional EBSD result of the USSR sample and shows a gradient structure. The grains in the surface layer are refined. The KAM values in the surface layer are significantly higher than those in the matrix and gradually decrease with increasing depth, manifesting decreased defect density, as shown in Figure 3(b). According to the KAM map, the gradient layer has a depth of approximately 300 *μ*m. To further characterize the microstructure of the USSR sample, high-magnification EBSD observation is conducted on the 10 *μ*m thick surface layer, as shown in Figure 4. The BC and IPF maps demonstrate that the ferrite grains separated by high angle grain boundaries (HAGBs) are refined to approximately 1.5 *μ*m and contain many nanoscale substructures. Most substructure boundaries exhibit a misorientation range of 2-15°, indicating that they are LAGBs, as shown in Figures 4(b) and 4(c), while the misorientations of some substructure boundaries are less than 2°, indicating that these boundaries belong to dense dislocation walls (DDWs). Therefore, the observed nanoscale substructures are composed of subgrains and dislocation cells.

TEM observation was further performed to reveal the detailed microstructure of the topmost surface layer, as depicted in Figure 5. The TEM images and the selected area electron diffraction (SAED) pattern confirm that the large ferrite grains are separated by many substructures composed of subgrains and a small number of dislocation cells. Many dislocations are still visible within these substructures. A small number of nanograins are visible. The average size of the substructures is 309.4 nm. Based on the EBSD and TEM observation, a GNS surface layer is formed in the USSR sample.

Figure 6 presents the variation of microhardness along an increasing depth of the investigated samples. The as-received sample has an almost invariable hardness along its depth. A gradually decreased microhardness is observed from the one USSR-treated surface to the matrix in the USSR sample, which results in a U-shaped hardness profile. The gradient hardness profile must be, in our view, a result of the gradient nanostructure. The thickness of the gradient layer is estimated to be 300 *μ*m from the hardness profile, which is consistent with EBSD observations.

Figure 7 presents the typical engineering stress-strain curves of the as-received and USSR samples. The as-received sample has a yield strength of 379.7 ± 15.0 MPa, an ultimate tensile strength of 527.3 ± 14.7 MPa, and an elongation of 0.36 ± 0.02. The USSR sample exhibits a yield strength of 474.9 ± 7.1 MPa, an ultimate tensile strength of 551.4 ± 10.1 MPa, and an elongation of 0.32 ± 0.001. This means that the yield strength of the USSR sample improves by 25.1% and is accompanied by a slightly reduced ductility.

## 4. Discussions

### 4.1. Strengthening Mechanism

Through our microstructure characterization, substructure boundary strengthening, grain boundary strengthening, dislocation strengthening, and hetero-deformation-induced (HDI) strengthening are identified as responsible for the high strength of the GNS surface layer. The GNS surface layer is mainly composed of the nanoscale substructures, which are very different from the nanograined structure in previous GNS which involves a large fraction of HAGBs [24–26]. The substructures are mainly separated by LAGBs and DDWs. These substructure boundaries can hinder dislocation motion like HAGBs, while their barrier effect is weaker than the latter due to their small misorientation (<2°). Therefore, the substructure boundaries have a relatively weaker strengthening effect, but less sacrificed ductility, which explains the origin of the high strength and good ductility of the USSR sample to a certain extent. The strengthening contribution of LAGBs *σ*_LAGB_ can be estimated using Taylor strengthening effect related to the average misorientation [27, 28]:

(1) $$\begin{array}{c} \sigma_{\text{LAGB}}=M\alpha Gb\sqrt{\rho_{0}+\frac{3f{\bar{\theta }}_{\text{LAGB}}}{bd}}, \end{array}$$

where *M* is the Taylor factor (3.06) and *α* is a constant (0.25). *G* represents the shear modulus and 80 GPa for steel [29], and *b* is the modulus of the Burgers vector of the gliding dislocation (0.25 nm for steel [29]). *ρ*_0_ is the dislocation density between the boundaries and less than 10^12^ [28]. ${\bar{\theta }}_{\text{LAGB}}$, *f*, and *d* present the average misorientation, fraction, and boundary space of LAGBs, respectively, which can be extracted from the EBSD data. Based on our EBSD result of the 10 *μ*m thick surface layer (Figure 4), *σ*_LAGB_ is as high as 490.58 MPa in this topmost surface layer. The grains separated by HAGBs in the GNS surface layer are slightly refined, thus contributing to enhanced strength through the grain boundary strengthening effect. However, this contributor is relatively small because the grain refinement is not obvious. The GNS surface layer also involves a high density of dislocations (Figures 3–5), which also contributes to strength improvement by obstructing dislocation motion. As a type of heterostructured material [30, 31], GNSs can induce an HDI-strengthening effect through mechanical incompatibility. The GNS also provides extra work hardening capacity, i.e., HDI hardening, which is regarded as the primary source origin of high ductility [32].

### 4.2. Formation of the GNS Surface Layer

Our microstructure characterization shows that the microstructure of the GNS layer is featured by refined grains, subgrains, dislocation cells, and dense dislocations, and no deformation twins are observed. Hence, the plastic deformation of the Q345 steel is mediated by dislocation activation. Based on previous literature [33, 34], it is suggested that the microstructure refinement of the Q345 steel induced by the USSR is operated through dislocation subdivision, which facilitates the formation of the GNS surface layer. During USSR processing, massive dislocations are activated to accommodate plastic strain and gradually develop DDWs. Prevailing DDWs subdivide the original ferrite grains into individual dislocation cells. Increasing plastic strain, DDWs gradually evolve into LAGBs through dislocation annihilation and rearrangement, leading to the formation of subgrains. Further increasing plastic strain, LAGBs transform into HAGBs, giving rise to grain refinement. This grain refinement process is similar to pure Fe and ferrite in other steels [33, 34]. Here, one pass of the USSR is performed with a relatively small static force, leading to small plastic deformation. Therefore, the substructures but not nanograins are prevailing in the GNS surface layer. More systematic experiments are needed to reveal the relationship between the process parameters of the USSR and the microstructure.

## 5. Conclusions

In the present work, a GNS surface layer is prepared on a commercial Q345 structural steel through one pass of the USSR. Nanoscale substructures composed of subgrains and dislocation cells are formed at the topmost surface layer. The GNS surface layer has a thickness of approximately 300 *μ*m. The uniaxial tensile measurement indicates that the yield strength of the USSR sample improves by 25.1% compared to the as-received sample, with a slightly decreased ductility. The nanoscale substructure, refined grains, high density of dislocations, and HDI strengthening are identified to be responsible for the enhanced strength of the USSR sample.

## Figures and Tables

**Figure 1:** The OM (a, b) and SEM (c, d) images of the as-received sample.

**Figure 2:** The EBSD result of the as-received sample: (a) IPF map, (b) grain size statistics, (c) BC map, and (d) KAM map. The black and white lines in (a, c) profile the HAGBs and LAGBs, respectively.

**Figure 3:** Cross-sectional EBSD result of the USSR sample: (a) IPF map and (b) KAM map. The black lines in (a) profile the HAGBs.

**Figure 4:** High-magnification EBSD result of the USSR sample in the topmost surface: (a) BC image, (b) misorientation change along the arrow in (a), (c) IPF map, and (d) KAM map. Black and white lines in (a, c) profile the HAGBs and LAGBs, respectively.

**Figure 5:** TEM images of the USSR sample in the topmost surface layer: (a, b) high-magnificent images and (c, d) low-magnificent images under (a, c) bright-field and (b, d) dark-field models.

**Figure 6:** Variation of microhardness along the increasing depth of the as-received and USSR samples.

**Figure 7:** Engineering stress-strain curves of as-received and USSR samples.

## Data Availability

Data is available on request.
